The article "Testis developmental related gene 1 promotes non-small-cell lung cancer through the microRNA-214-5p/Krüppel-like factor 5 axis" was retracted in 2024. Reasons: original data or images not available; unreliable results or conclusions; concerns about the data; concerns about the results or conclusions.

# Testis developmental related gene 1 promotes non-small-cell lung cancer through the microRNA-214-5p/Krüppel-like factor 5 axis

**DOI:** 10.1080/21655979.2021.2012406

**Published:** 2021-12-27

**Authors:** Xudong Lu, Nian Zhao, Guangjun Duan, Zhiyong Deng, Yimin Lu

**Affiliations:** a Soochow University, Suzhou, Jiangsu, China; b Department of Pulmonary and Critical Care Medicine, Affiliated Kunshan Hospital of Jiangsu University, Kunshan, Jiangsu, China; c Department of Science and Technology, Affiliated Kunshan Hospital of Jiangsu University, Kunshan, Jiangsu, China

**Keywords:** TDRG1, miR-214-5p, KLF5, NSCLC

## Abstract

Non-small-cell lung cancer (NSCLC) is a frequent malignancy and has a high global incidence. Long noncoding RNAs (lncRNAs) are implicated in carcinogenesis and tumor progression. LncRNA testis developmental related gene 1 (TDRG1) plays a pivotal role in many cancers. This study researched the biological regulatory mechanisms of TDRG1 in NSCLC. Gene expression was assessed by reverse transcriptase quantitative polymerase chain reaction (RT–qPCR). Changes in the NSCLC cell phenotypes were examined using 5-ethynyl-2ʹ-deoxyuridine (EdU), cell counting kit-8 (CCK-8), wound healing, flow cytometry, and Transwell assays. The binding capacity between TDRG1, microRNA-214-5p (miR‑214-5p), and Krüppel-like factor 5 (KLF5) was tested using luciferase reporter and RNA immunoprecipitation (RIP) assays. In this study, we found that TDRG1 was upregulated in NSCLC samples. Functionally, TDRG1 depletion inhibited NSCLC cell growth, migration, and invasion and accelerated apoptosis. In addition, TDRG1 interacted with miR-214-5p, and miR-214-5p directly targeted KLF5. The suppressive effect of TDRG1 knockdown on NSCLC cellular processes was abolished by KLF5 overexpression. Overall, TDRG1 exerts carcinogenic effects in NSCLC by regulating the miR-214-5p/KLF5 axis.

## Introduction

As a commonly diagnosed malignancy, non-small-cell lung cancer (NSCLC) has a high incidence [1]. NSCLC worsens considerably after metastasis by rapidly spreading to other body parts and organs, such as bone, liver and brain [2]. Some studies have suggested that NSCLC occurs more frequently in patients who have undergone heart or lung transplant surgery or those with a long smoking history, especially in advanced-age patients [3,4]. Despite great breakthroughs in NSCLC treatment, the therapeutic effect for advanced NSCLC patients remains unsatisfactory, and the five-year survival rate is merely 18% [5,6]. Therefore, developing novel therapeutic treatments is essential for prolonging NSCLC patients’ lives and helping to alleviate their suffering from the effects of cancer and related treatments.

Long noncoding RNAs (lncRNAs), made up of over 200 nucleotides, are unable to be translated into proteins and are regarded as regulatory molecules [7]. Many lncRNAs have been identified to regulate tumorigenesis in cancers in recent years. For example, lncRNA epidermal growth factor receptor-antisense RNA 1 facilitates squamous cell carcinoma cell invasion and migration by sponging miR-145 [8]. The knockdown of lncRNA deleted in lymphocytic leukemia 1 plays an inhibitory role in renal cell carcinoma [9]. Accumulating evidence shows that lncRNAs act as important regulators in NSCLC progression. For example, Kinectin 1‑antisense RNA 1 silencing inhibits NSCLC cell proliferation, increases apoptosis, and blocks tumor growth in nude mice [10]. HOXB cluster antisense RNA 3 exacerbates malignant phenotypes of NSCLC cells [11]. Furthermore, recent papers have demonstrated that lncRNA testis developmental related gene 1 (TDRG1) can be a carcinogenic molecule in cancers. TDRG1 enhances cervical cancer cell growth by upregulating mitogen-activated protein kinase 1 [12]. TDRG1 increases cell viability and migration in endometrial carcinoma [13]. Increasing evidence suggests that lncRNAs serve as competing endogenous RNAs (ceRNAs) to modulate the level of tumor‐related genes by binding to microRNAs (miRNAs) [14,15]. Moreover, a study demonstrated that TDRG1 silencing inhibits the growth and metastatic ability of NSCLC cells by regulating the miR‐873‐5p/zinc finger e‐box binding homeobox 1 axis [16].

In this study, we further sought to elucidate the molecular mechanisms of TDRG1 in NSCLC. Given its high expression in NSCLC, we hypothesized that TDRG1 may promote NSCLC progression by binding to miRNAs through the ceRNA pattern. We investigated the influences of TDRG1 on cell proliferation, invasion, migration, and apoptosis in NSCLC cells. In addition, the oncogenic mechanism of TDRG1 in NSCLC was also demonstrated. This study may provide new insights for the understanding of TDRG1 in NSCLC.

## Materials and methods

### Tissue samples

NSCLC tissues (n = 40) and adjacent nontumor lung tissues (n = 40) were obtained from NSCLC patients undergoing surgery at the Affiliated Kunshan Hospital of Jiangsu University. The collected samples were frozen in liquid nitrogen. Neither radiotherapy nor chemotherapy was performed on the patients before the surgery. No patients had infectious diseases or histories of treatment aimed at NSCLC. Informed consent was obtained from all participants. The protocol was approved by the Ethics Committee of Affiliated Kunshan Hospital of Jiangsu University.

### Cell culture

NSCLC cells (A549, H1299, LC-2/ad, GLC-82 and H520) and the normal lung cell line MRC-5 were purchased from the American Type Culture Collection (Manassas, VA, USA). Cells were then maintained at 37°C in Dulbecco’s modified Eagle’s medium (DMEM; Gibco, USA) containing 10% fetal bovine serum (Gibco) at 37°C in a humidified incubator with 5% CO_2_.

### Cell transfection

TDRG1 was knocked down by specific short hairpin RNAs designated sh-TDRG1#1/2, with control shRNA (sh-NC) used as a negative control. For overexpression of miR-214-5p, miR-214-5p mimics and the control (NC mimics) were constructed. KLF5 was overexpressed by pcDNA3.1 integrated with Krüppel-like factor 5 (KLF5 complete sequence, designated pcDNA3.1/KLF5, with empty pcDNA3.1 used as a control). It is likely that TDRG1 expression was upregulated by inserting its full length into the pcDNA3.1 vector. Transfection was performed using Lipofectamine 2000 (Invitrogen, Carlsbad, CA, USA) for 48 h. All plasmids were commercially provided by GenePharma (Shanghai, China). Cells were seeded in 24-well plates at 2 × 10^5^ cells/well, transfected with 40 nM shRNA vector or 0.2 μg overexpression vector following the instructions provided with the Lipofectamine 2000 (Invitrogen) as described previously [17], and harvested at 48 h for further analysis.

### Reverse transcriptase quantitative polymerase chain reaction (RT–qPCR)

Total RNA was extracted with TRIzol reagent (Invitrogen). Subsequently, an Omniscript RT Kit (Takara, Dalian, China) was used for reverse transcription. RT–qPCR was performed using SYBR Premix Ex Taq (TAKARA, Osaka, Japan) with a 7900HT Fast Real-Time System (ABI Company, USA). The 2^−ΔΔCt^ method was used to analyze the expression of TDRG1, miR-214-5p, and KLF5 [18]. U6 served as the normalization control for miR-214-5p expression, while glyceraldehyde-3phosphate dehydrogenase (GAPDH) served that role for TDRG1 and KLF5 expression. The sequences of the PCR primers are shown in Table 1.

**Table 1.** Primer sequences used for RT-qPCR

Target	Primer sequences (5′-3′)
TDRG1	Forward: CTGACTCTTTCCGTGAACG
TDRG1	Reverse: GGGATGGATCTTCCTAAGGG
miR-214-5p	Forward: TCTCTTGCTATAGAAGCACAAC
miR-214-5p	Reverse: TCCTCCACAATCATGCTGTGT
miR-1252-5p	Forward: TGTGAGGTGTAGAAAGAAGGAA
miR-1252-5p	Reverse: ATTAAGCTCATTTGGAATTCTCT
miR-873-5p	Forward: GCAGGAACUUGUGAGUCUCCU
miR-873-5p	Reverse: AGGAGACUCACAAGUUCCUGC
SOX4	Forward: CAAGATCATGGAGCAGTCG
SOX4	Reverse: GTCTTTGAGCAGCTTCCAG
PPTC7	Forward: CCTATGACCCAAATTATATGTCACC
PPTC7	Reverse: TCATCTGGCTTTCCACCTC
ZFAND5	Forward: AGAGCCAGTTGTCACTCAG
ZFAND5	Reverse: GTTTGGGCAATTCAGGAGC
KLF5	Forward: CTACTGCGATTACCCTGGT
KLF5	Reverse: GTGTGAGTCCTCAGGTGAG
DPYSL3	Forward: ATCATGCTGGAAGATGGCA
DPYSL3	Reverse: CAGGTCTGCCATCTTCCTC
JAG1	Forward: CCTGTGAAGTGATTGACAGC
JAG1	Reverse: CGTTGGAGGAAATATACCGC
E2F2	Forward: CAACTTTAAGGAGCAGACAGTG
E2F2	Reverse: CAGGTTGTCCTCAGTCCTG
PPM1A	Forward: GAAACCAAATGAAGAGGATGTG
PPM1A	Reverse: CCTCTAGGTCTAGTCATAAATCTG
ROCK1	Forward: GCAAACAGCATGCTAACCA
ROCK1	Reverse: CCAGTTTATATTCTTCCTCTGCC
POU2F2	Forward: AGACACTAATCATCAGAACCC
POU2F2	Reverse: AGCCTTGATCTTTGTACTGG
CRY2	Forward: GCTGCGTTTACATTCTCGA
CRY2	Reverse: GAGACTGAAGTAGGAACCTCC
GAPDH	Forward: TCAAGATCATCAGCAATGCC
GAPDH	Reverse: CGATACCAAAGTTGTCATGGA
U6	Forward: GCTTCGGCAGCACATATACTAAAAT
U6	Reverse: CGCTTCAGAATTTGCGTGTCAT

### Western blotting

Western blotting was performed using a standard and established protocol as previously published [19]. The proteins were collected from NSCLC cells and quantified using a bicinchoninic acid kit (Pierce, Appleton, USA). Subsequently, the protein samples were separated with 10% sodium dodecyl sulfate–polyacrylamide gel electrophoresis and then transferred onto polyvinylidene difluoride membranes. After being blocked with 5% skim milk, the membranes were probed with primary antibodies (Abcam Inc., USA) labeled with fluorescein, followed by incubation with secondary antibodies (Abcam Inc.). An Odyssey infrared scanner (Li-Cor Bioscience, Lincoln, NE, USA) was used to detect the protein bands. The images of proteins were visualized with chemiluminescent reagent kits (Thermo Fisher Scientific, Waltham, MA, USA). Primary antibodies against the following proteins were used: cyclin A1 (ab13337); CDK2 (ab76146); Bcl-2 (ab32124); Bax (ab32503); GAPDH (ab9484); and KLF5 (ab137676).

### 5-ethynyl-2ʹ-deoxyuridine (EdU) assay

A549 and H1299 cells were seeded in 96-well plates (2 × 10^3^ cells/well). Next, 100 µl of EdU (50 µM/L, KeyGEN, Nanjing, China) was added to the plates for 2 h of incubation. Cells were fixed with 4% paraformaldehyde in phosphate-buffered saline for 30 min. Cell nuclei were subsequently stained with 4ʹ,6-diamidino-2ʹ-phenylindole and then observed with a fluorescence microscope (Leica, Nikon, Olympus, Zeiss) [20].

### Cell counting kit-8 (CCK-8) assay

As previously documented [21], the cells were plated in 96-well plates (5 × 10^3^ cells/well) and incubated for 24, 48, and 72 h. At each time point, 10 μl of CCK-8 solution (Kumamoto, Japan) was added to each well for 4 h of incubation. A microporous plate reader (Multiskan MK3, Thermo Fisher Scientific) at 450 nm was used to detect the results. The experiments were conducted 3 times independently.

### Wound healing and Transwell assays

In the cell migration and invasion assay, mitomycin was added to exclude the interference of cancer cell proliferation. The transfected cells were seeded in 6-well plates at 6 × 10^4^ cells/well. A 200 μl of sterile micropipette tip was utilized to make an artificial wound when cell confluence reached 95%. Then, the suspended cells were washed with phosphate-buffered saline. Wound closure was photographed with a phase-contrast microscope (Olympus Corporation, Tokyo, Japan) at 0 and 24 h and quantified with ImageJ software [22].

Transwell chambers (Corning Inc., Corning, NY, USA) were precoated with Matrigel. NSCLC cells (5 × 10^4^) in serum-free medium were added to the upper chamber. Then, 500 μl of DMEM containing 10% fetal bovine serum was added to the lower chamber. After 24 h, the cells were washed with phosphate-buffered saline, fixed with methanol (Sigma, St. Louis, MO, USA), and stained with 0.1% crystal violet. Cells were visualized with a light microscope (Olympus Corporation) [23].

### Flow cytometry-based assay

An annexin V-fluorescein isothiocyanate (FITC)/propidium iodide (PI) double-labeling staining kit (BD Biosciences, San Jose, CA, USA) was used in this assay. The procedure was performed as previously described [24]. The cells (2 × 10^5^/well) in 6-well plates were collected, washed twice with cold phosphate-buffered saline, and resuspended in 1 × binding buffer. Subsequently, cells were stained with 10 μl of annexin V-FITC for 15 min and 5 µl of PI for 10 min in the dark at room temperature. Cells were examined using a FACSCanto II flow cytometer (BD Biosciences). Analysis of flow cytometry data was performed using FlowJo version X.10.0.7–1 (FlowJo, LLC).

### Subcellular fractionation assay

To determine the localization of TDRG1 in NSCLC cells, NE-PER Nuclear and Cytoplasmic Extraction Reagents (Thermo Scientific, USA) were utilized to separate the nuclear and cytoplasmic fractions according to the manufacturer’s protocol. Total RNAs were isolated with TRIzol (Invitrogen). Finally, the TDRG1 level was detected by RT–qPCR.

### Luciferase reporter assay

The 3′‐UTR sequences of KLF5 containing binding sites for miR-214-5p and the complete sequence of TDRG1 were cloned into the pmirGLO vectors (Promega, Madison, WI, USA) to generate the KLF1-Wt vectors and TDRG1-Wt vectors. The mutant sequences were constructed to generate the TDRG1-Mut vectors and KLF1-Mut vectors. NC mimics or miR-214-5p mimics were cotransfected with these vectors into A549 and H1299 cells using Lipofectamine 2000 (Invitrogen). A luciferase detection kit (Promega) was applied to measure the luciferase activities after 48 h [25].

### RNA immunoprecipitation (RIP) assay

RIP was performed using a Magna RNA-Binding Protein Immunoprecipitation Kit (EMD Millipore, Billerica, MA, USA) [26]. At 90% confluence, cells were centrifuged at 4°C for 5 min at 1,000 × g, washed with precooled phosphate-buffered saline and lysed with radioimmunoprecipitation assay lysis buffer. Subsequently, the lysates were incubated for 10 min at 4°C with human Ago2 antibody (ab186733; Abcam; 5 µg) conjugated to magnetic beads, with IgG antibody (ab172730; Abcam; 5 µg) used as the control group. Samples were treated with Proteinase K for 30 min at 55°C with gentle agitation. Immunoprecipitated RNA was isolated using TRIzol. Coprecipitated RNAs were purified, identified, and analyzed with RT–qPCR.

### Statistical analysis

GraphPad Prism software 5.0 was utilized for statistical analysis. One-way analysis of variance or Student’s t test was used to evaluate differences among groups. The results are shown as the mean ± standard deviation. Linear correlation analysis was performed using Spearman’s correlation coefficient. The value of *p* < 0.05 was considered statistically significant. All experiments were repeated at least three times.

## Results

This study aimed to determine the functional role of TDRG1 in NSCLC. We also investigated the molecular mechanisms underlying the functional role of TDRG1 in NSCLC. Its upregulation was confirmed in NSCLC samples collected in this study. As revealed by functional experiments, TDRG1 served as an oncogenic molecule to promote the proliferation, invasion, and migration of NSCLC cells. In terms of the mechanism, TDRG1 upregulated KLF5 expression by sponging miR-214-5p. Overall, TDRG1 exerts carcinogenic effects in NSCLC by regulating the miR-214-5p/KLF5 axis.

### TDRG1 is upregulated in NSCLC

Before investigating the role of TDRG1, its level in NSCLC was measured. RT–qPCR results showed that TDRG1 was significantly upregulated in NSCLC tissues compared to normal tissues (*p* = 0.000) (Figure 1(a)). We next sought to examine whether TDRG1 expression correlates with the clinicopathological parameters of NSCLC patients. The median value of TDRG1 expression was used as the cutoff to divide the patients into high (n = 18) and low (n = 22) expression groups. As shown in Table 2, a high TDRG1 level was significantly related to tumor-node-metastasis (TNM) stage (*p* = 0.013) and lymph node metastasis (*p* = 0.004). As shown in Figure 1(b), the TDRG1 level in NSCLC cells (A549, H1299, LC-2/ad, GLC-82 and H520) was significantly higher than that in the normal lung cell line MRC-5 (*p* = 0.000).

**Table 2.** Correlation between TDRG1 expression and clinicopathological parameters of NSCLC patients

Parameters	TDRG1 expression		*P* value
	Low n = 22	High n = 18	
**Gender**			
Male	12	10	0.949
Female	10	8	
**Age**			
<60	7	5	0.781
≥60	15	13	
**Tumor diameter (cm)**			
≤5 cm	11	11	0.482
>5 cm	11	7	
**TNM stage**			
I/II	16	6	0.013
III/IV	6	12	
**Lymph node metastasis**			
Negative	15	4	0.004
Positive	7	14	
**Degree of differentiation**			
Well/moderate	9	9	0.565
Poor	13	9	
**Histology type**			
Adenocarcinoma	10	10	0.525
Squamous carcinoma	12	8	
*p < 0.05 is considered statistically significant. (Chi-squared test)

**Figure 1.** **TDRG1 is upregulated in NSCLC**. (a) RT–qPCR analysis was used to measure TDRG1 expression in NSCLC tissues (n = 40). (b) The expression of TDRG1 in the normal lung cell line MRC-5 and the NSCLC cell lines (A549, H1299, LC-2/ad, GLC-82 and H520) was measured by RT–qPCR. ***p < 0.01.

### Silencing TDRG1 hampers cell processes in NSCLC

To probe the biological function of TDRG1 in NSCLC, we conducted follow-up experiments. Sh-TDRG1#1/2 was used to knock down TDRG1. The results indicated that TDRG1 was stably knocked down by sh-TDRG1#1/2, and sh-TDRG1#1, which had a higher transfection efficiency, was used for the subsequent experiments (*p* = 0.000) (Figure 2(a)). CCK-8 and EdU assays showed that in cells transfected with sh-TDRG1#1, cell viability (*p* = 0.002) and proliferation (*p* = 0.000) was significantly hampered (Figure 2(b-c)). Moreover, the cell apoptosis rate was increased in sh-TDRG1#1-transfected NSCLC cells, as demonstrated by flow cytometry (*p* = 0.000) (Figure 2(d)). Western blot analysis showed decreased protein expression of cyclin A1, CDK2 and Bcl-2 and elevated expression of Bax in A549 and H1299 cells after sh-TDRG1#1 treatment (Figure 2(e)). Furthermore, the wound healing results indicated that TDRG1 deficiency decreased the migration of NSCLC cells (*p* = 0.000) (Figure 2(f)). As revealed by Transwell assay, TARG1 knockdown induced a marked decrease in the invasion ability of NSCLC cells (*p* = 0.006) (Figure 2(g)).

**Figure 2.** **TDRG1 knockdown inhibits NSCLC cell processes**. (a) RT–qPCR was used to measure the transfection efficiency of sh-TDRG1#1/2. (b-c) The effect of TDRG1 silencing on NSCLC cell proliferation was assessed by CCK-8 and EdU assays. (d) Cell apoptosis after sh-TDRG1#1 transfection was determined by flow cytometry. (e) The levels of cyclin A1, CDK2, Bax and Bcl-2 in the sh-TDRG1#1 and sh-NC groups were assessed by Western blotting. (f-g) The migration and invasion abilities of TDRG1-silenced cells were tested by wound healing and Transwell assays. **p < 0.01, ***p < 0.01.

### Overexpression of TDRG1 promotes cell processes in NSCLC

Next, we explored the effect of overexpressed TDRG1 in NSCLC. The pcDNA3.1 was transfected into NSCLC cells. RT–qPCR results showed that TDRG1 was significantly upregulated after transfection (*p* = 0.000) (Figure 3(a)). Upregulated TDRG1 facilitated cell proliferation (*p* = 0.007) (Figure 3(b-c)). Moreover, cell apoptosis was promoted after overexpressing TDRG1 (*p* = 0.007) (Figure 3(d)). Western blot analysis showed upregulated protein expression of cyclin A1, CDK2 and Bcl-2 and downregulated expression of Bax in TDRG1-overexpressing cells (Figure 3(e)). Furthermore, TDRG1 significantly increased the migration and invasion of cells (*p* = 0.074) (Figure 3(f-g)). These results demonstrated the oncogenic properties of TDRG1 in NSCLC.

**Figure 3.** **TDRG1 promotes NSCLC cell processes**. (a) RT–qPCR was used to measure the transfection efficiency of pcDNA3.1/TDRG1. (b-c) The effect of upregulated TDRG1 overexpression on cell proliferation was determined by CCK-8 and EdU assays. (d) Cell apoptosis was assessed by flow cytometry. (e) The levels of cyclin A1, CDK2, Bax and Bcl-2 after TDRG1 overexpression were measured by Western blotting. (f-g) Cell migration and invasion in TDRG1-overexpressing cells were tested by wound healing and Transwell assays. *p < 0.05, **p < 0.01, ***p < 0.01.

### TDRG1 sponges miR-214-5p

Numerous investigations have suggested that lncRNAs in the cytoplasm act as ceRNAs by sponging miRNAs to control target mRNAs. A subcellular fractionation assay and RT–qPCR analysis revealed a higher proportion of TDRG1 in the cytoplasm of cells compared with that in the nucleus (Figure 4(a)). starBase was used to search for the potential miRNAs of TDRG1, and miR-214-5p, miR-1252-5p and miR-873-5p were discovered (search category: pancancer types: 1 cancer type). Subsequently, the RT–qPCR results indicated that miR-214-5p had a significantly low expression in NSCLC cells (*p* = 0.000) (Figure 4(b)). Therefore, miR-214-5p was selected for the subsequent experiments. MiR-214-5p was significantly upregulated after transfection with miR-214-5p mimics (*p* = 0.000) (Figure 4(c)). The binding site between TDRG1 and miR-214-5p is presented (Figure 4(d)). To validate the interaction of TDRG1 with miR-214-5p, we conducted luciferase reporter and RIP assays. As observed, miR-214-5p mimics greatly impeded the luciferase activity of TDRG1-Wt vectors and did not affect that of TDRG1-Mut vectors (*p* = 0.001) (Figure 4(e)). In addition, the enrichment of TDRG1 and miR-214-5p was detected in the Ago2 antibody group (*p* = 0.000) (Figure 4(f)). Moreover, TDRG1 was negatively related to miR-214-5p in NSCLC tissues (Figure 4(g)).

**Figure 4.** **TDRG1 sponges miR-214-5p**. (a) The proportion of TDRG1 expression in the nucleus or cytoplasm was assessed by subcellular fractionation assay and RT–qPCR. (b) The expression of predicted miRNAs in NSCLC cells was determined by RT–qPCR. (c) RT–qPCR was used to measure the efficiency of miR-214-5p mimics in A549 and H1299 cells. (d) The binding site of miR-214-5p on the TDRG1 sequence. (e-f) Luciferase reporter and RIP assays were used to detect the interaction between miR-214-5p and TDRG1 in NSCLC cells. (g) The correlation between TDRG1 and miR-214-5p expression in NSCLC tissues. **p < 0.01, ***p < 0.01.

### KLF5 is directly targeted by miR-214-5p

Four online tools, microT, miRmap, PicTar and TaretScan, predicted the targets of miR-214-5p. The data showed 11 possible mRNAs that may bind to miR-214-5p (Figure 5(a)). After overexpressing miR-214-5p, we found that only KLF5 was significantly downregulated (*p* = 0.002) (Figure 5(b)). Next, we observed that KLF5 expression was high in NSCLC tissues (*p* = 0.000) (Figure 5(c)). Importantly, we discovered that both knockdown of TDRG1 and upregulation of miR-214-5p downregulated KLF5 in NSCLC cells (*p* = 0.001) (Figure 5(d)). The binding site between KLF5 and miR-214-5p is shown (Figure 5(e)). In the luciferase reporter assay, significant attenuation of KLF5-Wt luciferase activity was observed in cells after miR-214-5p overexpression, while the luciferase activity of KLF5-Mut remained unchanged (*p* = 0.000) (Figure 5(f)). Additionally, a negative expression correlation between miR-214-5p and KLF5 and a positive expression correlation between KLF5 and TRGD1 in NSCLC tissues were observed (Figure 5(g)).

**Figure 5.** **KLF5 is targeted by miR-214-5p**. (a) The candidate mRNAs predicted in starBase are presented as a Venn diagram. (b) Expression of the predicted candidate mRNAs in miR-214-5p-overexpressing cells was measured by RT–qPCR. (c) RT–qPCR was used to measure KLF5 expression in NSCLC tissues. (d) The expression of KLF5 in cells transfected with sh-TDRG1#1 or miR-214-5p mimics was measured by RT–qPCR. (e) The binding site between KLF5 and miR-214-5p. (f) The interaction between miR-214-5p and KLF5 was confirmed by luciferase reporter assay. (g) The expression correlation between KLF5 and TDRG1 (or miR-214-5p) in NSCLC tissues. **p < 0.01, ***p < 0.01.

### The TDRG1/miR-214-5p/KLF5 axis modulates NSCLC cellular processes

Rescue assays were performed to further investigate the ceRNA network in NSCLC. As shown, transfection of sh-TDRG1#1+ pcDNA3.1/KLF5 recovered the reduction in KLF5 mRNA and protein expression induced by sh-TDRG1#1 (*p* = 0.000) (Figure 6(a)). Furthermore, the weakened cell proliferation ability caused by the transfection of sh-TDRG1#1 was enhanced after transfection with sh-TDRG1#1+ pcDNA3.1/KLF5 in NSCLC cells (*p* = 0.008) (Figure 6(b-c)). Additionally, the apoptosis of cells was elevated by sh-TDRG1#1, but this effect was abrogated by pcDNA3.1/KLF5 (*p* = 0.015) (Figure 6(d)). In addition, the TDRG1 knockdown-induced effect on cyclin A1, CDK2, Bax and Bcl-2 protein expression was reversed by overexpression of KLF5 (Figure 6(e)). As revealed in Figure 6(f-g), KLF5 upregulation abrogated the inhibitory effect mediated by TDRG1 silencing on cell migration and invasion (*p* = 0.016). Therefore, the TDRG1/miR-214-5p/KLF5 axis was involved in NSCLC cellular processes.

**Figure 6.** **TDRG1 modulates NSCLC cellular processes through KLF5**. (a) The levels of KLF5 mRNA and protein in A549 and H1299 cells transfected with sh-TDRG1#1 or sh-TDRG1#1+ pcDNA3.1/KLF5 were measured by RT–qPCR and Western blotting. (b-c) CCK-8 and EdU assays were performed to assess cell proliferation in the sh-NC, sh-TDRG1#1 and sh-TDRG1#1+ pcDNA3.1/KLF5 groups. (d) Apoptosis in the sh-NC, sh-TDRG1#1 and sh-TDRG1#1+ pcDNA3.1/KLF5 groups was determined by flow cytometry. (e) The levels of cyclin A1, CDK2, Bax and Bcl-2 after TDRG1 overexpression were measured by Western blotting. (f-g) The invasion and migration abilities of A549 and H1299 cells transfected with sh-NC, sh-TDRG1#1 or sh-TDRG1#1+ pcDNA3.1/KLF5 were evaluated by Transwell and wound healing assays. *p < 0.05,**p < 0.01, ***p < 0.01.

## Discussion

NSCLC has a high incidence of complications, and the postoperative survival rate of NSCLC patients is low [27]. LncRNAs have been confirmed in many studies as important participants in cancer progression [9,28]. LncRNA TDRG1 has also been reported to accelerate the development of many malignancies [12,13]. In this research, we discovered that TDRG1 was overexpressed in NSCLC tissues and cells. Moreover, TDRG1 depletion reduced cell proliferation, migration, and invasion and increased apoptosis. These findings confirmed the oncogenic role of TDRG1 in NSCLC.

Furthermore, studies on ceRNA networks have been widely reported in recent years. LncRNAs serve as molecular sponges for miRNAs to influence mRNA expression levels and thereby affect the process of cancers [29–32]. Additionally, TDRG1 participates in the progression of cancers as a ceRNA. For instance, TDRG1 competes with human fibroblast growth factor for sponging miR-873-5p to accelerate the development of gastric carcinoma [33]. As an oncogene, TDRG1 enhances the proliferation of cervical cancer cells by sponging miR-330-5p to upregulate an ETS domain-containing protein [34]. In this research, it was predicted that TDRG1 contains a binding site for miR-214-5p. MicroRNAs (miRNAs), a kind of small ncRNA, are widely reported as regulators in multiple biological processes [35]. Moreover, the role of miR-214-5p in many cancers has been elucidated. For example, miR-214-5p regulates collapsin response mediator proteins to inhibit cell proliferation in prostate cancer [36]. MiR-214-5p suppresses cell invasion and migration in hepatocellular carcinoma [37]. Here, it was confirmed that miR-214-5p was downregulated in NSCLC cells. Additionally, TDRG1 was proven to interact with miR-214-5p and to be negatively related to miR-214-5p. We concluded that TDRG1 acts as a sponge of miR-214-5p.

Furthermore, we identified that Krüppel-like factor 5 (KLF5) was targeted by miR-214-5p in NSCLC cells. KLF5 contributes to cervical cancer by upregulating expression of tumor necrosis factor receptor superfamily member 11a [38]. KLF5 exacerbates thyroid cancer by activating nuclear factor κB signaling [39]. Moreover, KLF5 was reported to be overexpressed in NSCLC and to play an oncogenic role [40,41]. Mounting evidence shows that miRNAs exert regulatory effects by regulating their target mRNAs in the progression of cancers, including NSCLC [41–43]. Moreover, it has been reported that miRNAs participate in tumor progression by targeting KLF5. MiR-145-5p facilitates gastric cancer by binding to the KLF5 3ʹ-UTR [44]. MiR-493-5p suppresses osteosarcoma cell proliferation by downregulating KLF5 [45]. Here, KLF5 was found to be upregulated in NSCLC tissues. We further confirmed that miR-493-5p targeted KLF5 and negatively regulated KLF5. Additionally, TDRG1 upregulated KLF5 expression by sponging miR-493-5p. Rescue assays demonstrated that overexpressing KLF5 rescued the inhibitory effect of TDRG1 silencing on the cellular development of NSCLC.

## Conclusion

In summary, this work validated the abnormal expression of TDRG1 in NSCLC tissues and cells and showed that TDRG1 functions as an oncogene in NSCLC to promote cell proliferation, migration, and invasion through the miR-214-5p/KLF5 axis. Therefore, our study suggested that TDRG1 may be a promising diagnostic biomarker and therapeutic target of NSCLC. In the future, we will conduct in vivo experiments to further confirm the role and mechanism of TDRG1 in NSCLC.

## Limitation

The present study is not without limitations. First, the clinical sample size of the NSCLC patients should be increased to further verify the clinical significance of our findings. Second, the related signaling pathways targeted by the TDRG1/miR-214-5p/KLF5 axis remain unclear and require further investigation.

## Supplementary Material

Supplemental Material

## Highlights

- TDRG1 is upregulated in NSCLC tissues and cell lines.
- TDRG1 overexpression contributes to malignant features of NSCLC cells.
- TDRG1 positively regulates KLF5 expression by sponging miR-214-5p.
- TDRG1 exerts carcinogenic effects in NSCLC by upregulating KLF5 expression.
